This article has been retracted.

# Collecting duct carcinoma of the kidney: a clinicopathological study of five cases

**DOI:** 10.1186/1746-1596-8-96

**Published:** 2013-06-17

**Authors:** Xiangyang Wang, Jianwei Hao, Ruijin Zhou, Xiangsheng Zhang, Tianzhong Yan, Degang Ding, Lei Shan, Zhonghua Liu

**Affiliations:** 1 Department of Urology, Henan Provincial People’s Hospital, Zhengzhou 450003, China

**Keywords:** Renal tumor, Collecting duct carcinoma, Diagnosis, Pathology

## Abstract

**Objective:**

To investigate the clinicopathological features of collecting duct carcinoma (CDC) and improve its diagnosis and treatment.

**Methods:**

A retrospective analysis was performed with clinical data including follow-up results of five patients with CDC.

**Results:**

A total of 5 cases, including 4 males and 1 female, were included in this analysis with the average age 54 years (range 42 to 65). Patients mainly suffered from lumbar pain, hematuria, abdominal mass and low grade fever. Four patients underwent radical nephrectomy while another received palliative nephrectomy. Lymph node metastasis occurred in 3 cases and renal hilum fat metastasis happened to 2 other cases. Tumors was located in the renal medulla and presented invasive growth. They had a tubulopapillary architecture with the hobnail-shaped cells protruding into the glandular lumen, and were accompanied by interstitial fibrosis and dysplasia of epithelial cells in collecting ducts adjacent to the tumors. One tumor was staged at AJCC II, two at AJCC III and two at AJCC IV. Postoperative interferon immunotherapy was applied in 2 cases. Patients were followed up for 5 to 18 months and the average survival time was 10 months.

**Conclusion:**

The CDC exhibits special clinicopathological features, high degree of malignancy and poor prognosis. The diagnosis depends on the histopathological examination. Early detection and early surgical treatment are still the main methods to improve the prognosis of patients with CDC.

**Virtual Slides:**

The virtual slide(s) for this article can be found here: http://www.diagnosticpathology.diagnomx.eu/vs/3702794279387989

## Background

Collecting duct carcinoma (CDC) is a type of kidney cancer that originates in the duct of Bellini of the kidney and also known by several synonyms like Bellini duct carcinoma, medullary renal carcinoma, distal renal tubular carcinoma and distal nephron carcinoma [1,2]. CDC is an unusual variant of renal cell carcinoma and accounts for about 1% of all renal cell carcinomas. CDC is differentiated from other renal cell carcinomas by its characteristic location, typical histological appearance and poor prognosis [1]. CDC metastasizes to regional lymph nodes in approximately 80% of cases, to the lung or adrenal gland in 25% and to the liver in 20% [3]. Average survival time has been reported to be 22 months [4]. Several treatments have been proposed but with limited efficacy, including radiation therapy, immunotherapy, chemotherapy, as well as combination therapy [4-6].

Although many relevant studies have been reported [7-9], it is necessary to gather more clinicopathological features of CDC to better diagnose and treat it. Therefore, we reported our experience with 5 CDC patients from August 2001 to September 2010 and explored their clinicopathological features and treatments in combination with literature review.

## Materials and methods

### Clinical data

Five patients (4 males and 1 female) with pathologically diagnosed CDC were included. The average age was 54 years (range 42 to 65). The tumors were found in the right kidneys in 3 cases and in left kidneys in 2 cases. Clinical manifestations included waist and abdomen pain in 4 cases, hematuria in 3 cases, low grade fever in 1 case, and local mass in 1 case. Extracorporeal shock wave lithotripsy was historically applied for 1 patient with ureteral stones. Accessory examinations revealed an increase in the levels of red blood cells and urine protein in 3 cases, elevated erythrocyte sedimentation rate in 3 cases, and negative results of urine cytology in all of 5 cases. Analyses by Color Doppler ultrasound and computerized tomography (CT) demonstrated that tumors were located in the center of kidney and near the pelvis; that invasion of renal hilum was observed in 2 cases, containing surrounding of tumor tissue on the renal artery in 1 case; that the diameter of tumors was between 4.6 and 10.5 cm with average 6.8 cm; and that hydrocalycosis was observed in 3 cases. Type-B ultrasonic examination found hypoechoic masses with ill-defined border in the central region around renal sinus as well as pelvis invasion of the mass in some cases (Figure 1). Magnetic resonance imaging (MRI) indicated isointensity on Tl-weighted images (T1WI) and hypointensity on T2WI in the renal sinus and confirmed caliectasis (Figure 2). Masses near the renal sinus were also detected by CT, which were further determined as slight or moderate, progressive, delayed enhancement by enhanced dynamic scanning (Figure 3).

**Figure 1:** **Ultrasound showing left renal tumor. A**: Ultrasound revealed hypoechoic masses (arrow) with ill-defined border in the central region around renal sinus. **B**: Color doppler flow imaging of mass (arrow) indicated decreased blood flow signals. The tumor invaded renal pelvis inward and infiltrated vessel pedicle outward, and caused caliectasis. AO: abdominal aorta; LRA: left renal artery.

**Figure 2:** **MRI showing the left renal tumor.** The mass in the left renal sinus showed homogeneous isointensity on T1WI (**A**, arrow) and hypointensity on T2WI (**B**, arrow).

**Figure 3:** **CT showing left renal tumor.** Plain CT scan revealed a heterogeneous density in the left renal tumor (**A**, arrow). The borders between the tumor and abdominal aorta, kidney and renal vein were not clear. Enhanced CT scan suggested a slight enhancement in the arterial phase (**B**, arrow) and a moderate enhancement in the venous stage (**C**, arrow).

### Clinical stages

WHO classification of renal carcinoma (2004) was chosen as the pathological diagnostic criteria, and TNM and clinical staging were conducted based upon the clinicopathological information of the cases and the criteria developed by American Joint Committee on Cancer (AJCC) in 2002.

### Treatment methods

Radical nephrectomy was applied to 4 cases. Palliative nephrectomy was applied to another case as the tumor tissues in this patient surrounded the renal artery and vein and integrated with multiple lymph nodes. Primary lesion tissues and Para-aortic lymph nodes were removed as much as possible. Postoperative immunotherapy was administered for 3 cases by subcutaneous administration of 9 million units of interferon-α each time (3 times a week and 12 weeks a cycle). Chemoradiotherapy was not given to any of the five cases.

## Results

### Pathological results

Visual examination indicated that the tumors were mainly found in the renal medulla, gray or yellow, showing necrosis or hemorrhage; they exhibited invasive growth with ill-defined border and no pseudocapsule (Figure 4A). Microscopical inspection suggested that tumor cells had a tubulopapillary architecture and formed hobnail pattern along the glandular tube. They also showed eosinophilic or basophils properties, ill-defined border, large nuclei, and prominent nucleoli, and were accompanied by interstitial connective tissue reaction. Primary CDC or dysplasia was seen in tissues around the tumors (Figure 4B, C, D, E and F). Renal hilar lymph node metastasis appeared in 3 cases. Immunohistochemical tests showed cytokeratin (CK) (+), peanut agglutinin (PNA) (+) and high-molecular-weight cytokeratin (CK34BE12) (+) in all of 5 cases, Vimentin (+) and epithelial membrane antigen (EMA) (+) in 4 cases, low molecular weight cytokeratins (CAM5.2) (+) and Ki67 (+) in 2 cases, and alpha-fetoprotein (AFP) (−), chromogranin A (CgA) (−), synaptopodin (SYN) (−), Villin (−) and Wilms' tumor gene 1 (WT1) (−) for all cases. TNM staging and clinical staging are shown in Table 1.

**Figure 4:** **Pathological examination. A**: The gray renal tumor without capsule. **B**: The tumor cells exhibiting a tubulopapillary architecture. **C**: Hobnail-shaped cells protruding into the glandular lumen (arrow). **D**: The tumor cells exhibiting eosinophilic property with ill-defined bound, large and atypical nuclei, and prominent nucleoli. **E**: The tumor interstitial connective tissue reaction. **F**: Collecting duct carcinoma in situ or dysplasia (indicated by an arrow).

**Table 1:** Staging and treatment outcomes of five collecting duct carcinoma patients

	**1**	**2**	**3**	**4**	**5**
Venous tumor thrombus	No	Yes	No	No	No
Lymphatic metastasis	No	No	1/8	5/6	3/4
Metastasis	No	No	No	Fat tissue in renal hilus	Fat tissue in renal hilus
TNM staging	T_2_N_0_M_0_	T_3b_N_O_M_O_	T_2_N_1_M_0_	T_4_N_2_M_0_	T_4_N_2_M_O_
AJCC staging	II	III	III	IV	IV
Operation	Radical nephrectomy	Radical nephrectomy	Radical nephrectomy	Palliative nephrectomy	Radical nephrectomy
Immunotherapy (IFN -α)	No	2 cycles	No	No	1 cycle
Survival time (month)	18	12	9	6	5

### Treatment outcomes

Multiple metastases to liver, vertebrae, lung and retroperitoneal happened to all 5 cases at 5–18 months after operation, and the average survival time was 10 months (Table 1).

## Discussions

CDC is located in the renal medulla and originates from the epithelial cells of Bellini collecting ducts [1]. Because of its unique biological and pathologic characteristics that are different from the other renal cell carcinomas, it’s considered to be an independent histological type. Currently, WHO names it as Bellini duct carcinoma [10].

CDC can occur at any age, and is more common in young adults. Men are more susceptible than women with the ratio of about 2:1. Tokuda et al. [11] report that the average onset age is 58 years and male patients account for 71.6% of the cases. In present study, the average age was 54 years. Common clinical symptoms of CDC include painless gross hematuria, lumbar abdominal pain, waist and abdominal mass, fatigue, fever, and weight loss. It has a short and fast course. Normally, metastasis occurs in most of patients before treatment, including bone metastasis and lymph node metastasis [11]. Three cases of lymph node metastasis and two cases of renal hilum fat metastasis were reported in the present study. Researchers have reported that CDC shows similar biological properties to those of urothelial cell carcinoma. Thus it is considered that they both originate from renal tubular and can occur simultaneously [12].

Imaging examinations are the main methods for CDC diagnosis. The tumors are hypo-vascular with ill-defined border, and pose invasions to the renal cortex and renal sinus [13,14]. Hydrocalycosis often occurs because of the extruding from the tumors. Color ultrasound can reflect a hypoechoic, homogeneous or heterogeneous mass with irregular morphology and ill-defined bounder, as well as reduced blood flow signal. CT is able to detect the invasions of tumors into pelvis and renal cortex. Calcification and hemorrhage can also be seen in some cases. Mild to moderate uneven delayed enhancement can be detected in dynamic contrast-enhanced scan [15]. MRI gives iso-intensity or hyper-intensity on T1WI and hypo-intensity on T2WI. The 5 cases in this study showed similar symptoms. CDC doesn’t have specific imaging features that distinguish it from other types of renal cell carcinoma such as renal medullary carcinoma, sarcomatoid renal cell carcinoma, and renal pelvis carcinoma, so its diagnosis requires pathological examination.

The pathological examination is the gold standard for diagnosis of CDC. As the tumors grow, they usually infiltrate into renal pelvis, renal cortex, and even renal hilum. CDC usually presents a tubulopapillary architecture, and tumor cells form hobnail pattern along the glandular tube. Poorly differentiated tumor cells show nest-shaped, rope-like, sarcomatoid or adenoid cystic morphology, with or without interstitial connective tissue reaction [15-17].

Kidney cancer can be classified as multiple types based on the origin of tumor cell types, including renal cell carcinoma (RCC, the most common type), tubulocystic renal carcinoma [18], renal solitary fibrous tumor [19], renal pigmented paraganglioma [20], and renal endocrine tumors [21]. In addition to histological analyses, genetical and biochemical approaches are becoming more and more important for the differentiation and diagnosis of renal carcinomas. Genetical analyses include gene copy numbers, chromosomal imbalances, gene mutations and single nucleotide polymorphism (SNP) analysis [18]. Many biomolecules, including epithelial-mesenchymal transition (EMT) markers such as N-cadherin [22] and vimentin [19] and human leucocyte molecules such as HLA-G and HLA-E [23], are reported to be biomarkers for renal cancer. Immunohistochemical examination of these biomarkers is important for the determination of the origin and the diagnosis of CDC. Cancer cell have positive expressions of CK (AE1/AE3), CK7, CK19, EMA, vimentin, CK34BE12, PNA and ulex europeus agglutinin (UEA), and negative expression of CD10 and CK20. Combination of CK34BE12 and PNA is able to detect 90% of CDC [24]. The results from pathological and immunohistochemical examinations are the important basis for the diagnosis of CDC and for differentiating it from other types of kidney cancer.

Radical nephrectomy is the major method to treat CDC. As the tumor cells spread in cortical collecting tubule, which results in poor prognosis, tumor enucleation and partial nephrectomy are not favorable. However, radiotherapy, chemotherapy and immunotherapy have limited efficacy on CDC [12]. The postoperative survival time for the 2 cases of stage IV was 5 to 6 months, 18 months for the case of stage II, and 9 to 12 months for the 2 patients of stage III. Therefore, early detection and early surgery are the best way to prolong the renal collecting duct carcinoma survival time. Recently, there are a few reports on the effectiveness of targeted therapy with Sunitinib and sorafenib in treatment of CDC [25-27]. However, there’s a study indicating no response of targeted therapy [17]. Therefore, the efficacy of targeted therapy on CDC remains to be demonstrated.

Overall, our reports are beneficial supplements for better understanding the clinicopathological features of CDC. At the same time, the treatments and corresponding outcomes are valuable information for guiding future clinical practice.

## Consent

Written informed consent was obtained from the patient for publication of this report and any accompanying images.

## Competing interests

The authors declare that they have no competing interests.

## Authors’ contribution

XYW and JWH participated in the design, analyses and data interpretation and drafted the manuscript. RJZ, XSZ, TZY, DGD, LS, and ZHL helped to retrieve pathologic and clinical information and provide valuable insight during manuscript preparation. All authors reviewed and approved the final manuscript.
